RETRACTED

# Analysis on Health Information Acquisition of Social Network Users by Opinion Mining: Case Analysis Based on the Discussion on COVID-19 Vaccinations

**DOI:** 10.1155/2021/2122095

**Published:** 2021-09-21

**Authors:** Datian Bi, Jingyuan Kong, Xue Zhang, Junli Yang

**Affiliations:** ^1^School of Management, Jilin University, Changchun 130022, China; ^2^School of Journalism and Communication, Jilin University of Finance and Economics, Changchun 130117, China

## Abstract

This study aims to explore phenomena and laws that occur when different users on social network platforms obtain health information by constructing an opinion mining model, analyzing the user's position on selected cases, and exploring the reflection of the phenomenon of truth decay on platforms. It selects group posts regarding the COVID-19 vaccination dispute on the Douban platform, analyzes the positions of different users, and explores phenomena related to users obtaining health information on domestic social platforms according to different topics and information behaviors. The results reveal a linear relationship between the negative and neutral attitudes of netizens on social networking platforms. Moreover, netizens tend to hold subjective language when expressing their views and attitudes, and their views on social platforms will not change easily. The study explores the health information acquisition behavior of netizens on social platforms based on the constructed user opinion mining model. The study is helpful for relevant units and platforms to make scientific decisions and provide guidance according to different positions of Internet users.

## 1. Introduction

With the popularity of the Internet and the widespread application of social media platforms, the speed and scope of netizens' access to information and communication have undergone tremendous changes. Currently, the Internet has become the fourth largest source of health information after mass media, health professionals, and family members. People are accustomed to searching for health information before and after medical consultation and expressing their own opinions for social interaction on social platforms. While this significant change has brought ease and convenience, it has also resulted in a mix of true and false information on social media platforms.

The parallel spread of truth and rumors makes it difficult for netizens to distinguish which information is authentic. In 2016, “post-truth” was selected as the word of the year by the Oxford Dictionary, and as the use of “fake news” sharply increased in 2017, the RAND Corporation of the United States started exploring the diminishing role of facts and analysis and launched “truth decay” on its 2018 report. Whether it is “post-truth,” “fake news,” or “truth decay,” these phases represent the difficulty to reach consensus and fuel the desire to question one another on social platforms. However, the Internet is bound to become even more important due to the various changes of types of Internet users and their information behavior; therefore, social platforms should aim at providing more reliable and accurate online health information in the near future.

RETRACTED

In view of this, this research builds a “COVID-19 vaccine” opinion analysis dictionary based on specific health information acquisition data, which counts the neutral, positive, and negative opinions of netizens and discusses hot topics based on user information behavior and netizen posts. To explore the truth decay that occurs when netizens obtain health information on social platforms, this paper provides more reference opinions for related platforms to monitor the dissemination of health information. The article is divided into six parts. The first introduces the background of this research, and the second summarizes the research results on health information and opinion mining in social platforms, introducing the concept of truth decay and its performance trends. The third introduces the model of point mining in this research and elaborates on the acquisition and processing of data. The fourth is based on the information behavior of netizens and their discussion topic words. The fifth discusses this article's research results. Finally, the limitations and shortcomings of this research are analyzed, and directions for future related studies are proposed.

## 2. Literature Background

### 2.1. Health Information Platform

Social media platforms have gradually become an important channel for netizens to obtain and share health-related information. New media, especially social network platforms, have great potential in supporting information search and decision-making on self-care and health-related issues [1]. Research shows that people's search for health-related information on the platform is based on trust; further, sharing and discussing topics related to health show different user behaviors on social platforms [2, 3]. In the past, people tended to ask friends and family for information and advice on how to deal with illness; now, netizens can exchange health information on a large number of virtual communities on social platforms [4]. This kind of digital health community not only helps people find more timely and personalized health-related information [5] but also helps patients discuss and share their medical experience to realize the exchange of personal health information on the platform [6]. Lin et al. [7] built an analysis model based on the data of users' health information exchange experience on Facebook and found that users' interaction behaviors can promote effective health information exchange; however, this kind of interaction behavior is significantly affected by health conditions. In other words, netizens are more inclined to share their health information when they are healthy [8].

RETRACTED

### 2.2. Opinion Mining

When netizens use the media to obtain health information, they also share health information through the platforms to propose opinions and behaviors that affect each other. Different attitudes and opinions on specific network events [9] or even opposing views have attracted many scholars in the domestic and foreign academic circles to use viewpoints to explore and conduct corresponding investigations [10]. Opinion mining means extracting people's opinions, emotions, evaluations, and attitudes and analyze emotions expressed on entities and their attributes from text information [11]. The current methods of opinion mining are mainly divided into two categories. The first category includes analyzing the characteristics of the text based on machine learning technology, and the LDA topic model can be used to identify public opinions in multiple dimensions [12]. Shallow machine learning techniques such as the Hidden Markov Model [13] and Conditional Random Fields [14] are used to extract users' evaluations. Liu et al. [15] used the Decision Tree Model to mine the vocabulary of diabetes risk in electronic medical records and found that this method can improve the accuracy of extracting opinions. With the continuous development of deep learning methods, different levels of depth of neural network models (CNN, RNN) can also express text as vectors to extract opinion attributes, which can mine opinion more efficiently and accurately in the network public opinion data of emergencies with complex relationships and arbitrary expressions [16]. Another type of method relies on the construction of a dictionary for opinion mining constructed by Hu et al. [17], which is based on the part of speech extraction of high-frequency words and uses nouns as the object of opinion evaluation and adjectives or verbs as opinion evaluation words. Taboada et al. [18] believe that the use of adjectives can better judge the text's position tendency, and weighting among different adjectives can extract the attributes of dictionary-based text opinion. The method based on sentiment dictionary is closer to human cognition, especially when combined with analysis mining algorithms, which is widely used in sentiment analysis.

RETRACTED

### 2.3. Truth Decay

In our living social environment, facts and data are vital to survival and are necessary conditions for success. Even if one must rely on subjectivity and intuition to make some complex decisions, these can also be confidently made through unanimous facts and reliable data. The innovation of new media technology and the different levels of human education have led to deviations at the cognitive level. Fake news ignores truthful sources, continues to spread on the Internet, and wantonly distorts the public's perception of the truth. At present, many scholars focus their research on the “post-truth era” and the discussion of the spread of “fake news,” but these discussions are not accurate. First, facts and data have always existed in society, but they have been selectively ignored in speeches, the increasing relative volume, and the resulting influence of opinion and personal experience over fact, disseminated by traditional and social media [19]. Second, “fake news” is fundamentally caused by changes in the way of human process information, economic conditions, and various changes in the current political and media environments. The root cause of people's distrust of data and objective facts cannot only be solved by preventing the release of fake news; accordingly, the RAND Corporation of the United States issued a report in January 2018, advancing the phase of “truth decay” to refer to the phenomenon by which people no longer believe in data and facts for decision-making but only rely on their own feelings after gathering facts and opinions. Thus, in this trend, the truth becomes increasingly less important. This erosion of trust and reliance on facts, data, and analysis involves many fields, such as public health, financial planning, and politics. It not only affects people's views on different events but also determines different decisions made by netizens.

Truth decay is mainly manifested in four trends. The first trend is that the increasing number of facts does not increase the public's recognition of them, but the public has its own views on the analysis and interpretation of facts and data. This trend is mainly concentrated on the divergence of two kinds of related information: (1) facts released by relevant authoritative medical institutions (e.g., new discoveries about the benefits of cancer treatment), though netizens are more willing to believe in smoking and cancer in response to this uncertain explanation (smoking can cause lung cancer, but netizens are more inclined to smoke to all cancers which may be related to smoking); (2) facts and opinions that are gradually blurred and often confused. Some of the most powerful examples of blurring the line between opinions and facts come from print and media news sources—for example, some established media use reports that combine opinions and facts when publishing news. This writing method can be misleading when people obtain information, and it makes it more difficult for them to analyze and extrapolate objective facts from the author's perspective. The third trend is that people tend to be more subjective and rely on personal experience when making decisions, and their view is more convincing than facts. The third trend is closely related to the fourth trend, by which the public's trust in previously respected information sources (such as mainstream media and the government) has declined, and the authenticity of news information proposed by authoritative organizations is questioned by the public. At present, the amount and type of information that people can obtain from new media platforms are completely different from those in the late 2000s. The rise of social media platforms has also played a role in the relative increase of dissemination across the information system. Although high-quality news and information are more readily available than ever before, there are also more trivial, one-sided, and false opinions. From a psychological point of view, people tend to believe in their own experiences and beliefs more than in disturbing facts, and advances in social media have exacerbated these trends.

RETRACTED

## 3. Data and Methodology

Although social networks provide platforms for netizens to express their opinions, exchange experiences, and promote the development of health information dissemination, lies, rumors, gossip, and other opinions circulate freely on the Internet under the guise of truth, which will cause the quality of health-related information on the platform to be uneven. Many statements are misleading and have no credible value information [20]. As COVID-19 swept the world, fake news and misinformation in social media have also followed, and it has become far more popular to spread such misleading posts than accurate information and public health-related reports about the disease [21]. The dissemination of false information on the platform will cause netizens not only to be unable to judge the authenticity of the information but also to generate many different opinions and positions, more seriously for endangering people's lives. In the past, the academic community has achieved corresponding results in terms of health information acquisition and related information behaviors in social platform communities; however, a few studies have explored the phenomenon of netizens on social media platforms in this kind of misinformation environment. This article thus selects a group of users on the Douban platform to discuss the topic of “COVID-19 vaccine injection (Hereinafter referred to as COVID-19 vaccination),” gathering the opinions of different users based on the method of opinion mining and analyzing the truth decay that occurs when users obtain health information in a fake news environment on domestic social platforms.

RETRACTED

### 3.1. Research Framework

The author of the RAND's report focused on issues related to presidential and congressman elections, the gap between the rich and the poor, racism, climate change, genetically modified foods, vaccine disputes, gun violence, gender discrimination, terrorism, and so on, and they discussed the manifestation of truth decay trend in American society. Hence, this study is based on this basic domestic situation, taking the topic of “vaccine dispute” as an example to explore the reflection of the truth decay of users' access to the health information on domestic social platforms. The research framework is shown in Figure 1.

Figure 1 presents the framework diagram of this article's reasoning. The study uses the method of opinion mining to conduct research on the acquisition of relevant health information on social media platforms. Moreover, based on the research method of case analysis, it selects the relevant topic of “vaccine dispute” in the Douban platform group as the analysis object, crawls the topic posts and user-related information behavior in the group discussion, and extracts all the comment text information separately to create a new text library.

### 3.2. Opinion Mining Model

To better explore the different opinions of netizens, we constructed a user opinion mining model. Firstly, we performed word segmentation on the text in the database and filters the meaningless and unrepresentative words in the vocabulary. The result was a comment vocabulary set (comment_*w*_), where *w* is the word representing the number of word segmentations of each comment. Then, we built two vocabularies as Negative = {N-word} and Positive = {P-word}. The former contained words expressing disagreement with or inability to get vaccinated. The latter contained words that agree with vaccination. Then, we found words containing positive and negative opinions and calculated the positive opinion index (pos · weight) and the negative opinion index (neg · weight) separately according to the position dictionary. We matched the vocabulary set of the text library with the negative vocabulary set and the positive vocabulary set and calculated the opinion position tendency of each comment. The calculation of the netizens' tendency to comment and stand is

(1) $$\begin{array}{c} \text{Score}=\sum \text{word}\in \text{Positive}-\sum \text{word}\in \text{Negative}. \end{array}$$

According to (1), the netizen's position score can be calculated, and according to the research of the position score index, the position of netizens can be represented by

(2) $$\begin{array}{c} \text{Score}=\left\{\begin{array}{cc} 1, & \text{If Score}>0\left({\text{Netizens}}^{\prime }\text{ views are positive}\right),\\ 0, & \text{If Score}=0\left({\text{Netizens}}^{\prime }\text{ views are neutral}\right),\\ -1, & \text{If Score}<0\left({\text{Netizens}}^{\prime }\text{ views are negative}\right). \end{array}\right. \end{array}$$

Formula (2) can be used to judge the opinions and positions of netizens' comments. A positive viewpoint means that netizens support or are willing to vaccinate, while a negative viewpoint means that netizens oppose or have negative feelings about the vaccine. A neutral viewpoint means that netizens have no obvious stance or reservations about vaccine injection. Finally, the research work also combined user information behavior and topic content to explore related phenomena in the process of users' health information acquisition on social platforms from different positions.

RETRACTED

### 3.3. Data Collection and Processing

Douban is a community platform that allows users to exchange views and opinions on books, movies, music, and other works, and it has developed a sharing community (Douban group). Douban has a large spontaneously formed group that generates hundreds of thousands of topics every day and gathers all kinds of people who can easily find the theme they like and a community of like-minded people. Netizens' discussions on the platform are not limited to books, movies, and music but also include entertainment, technology, humanities, photography, medicine, and many other fields. Douban has many features such as voting and provides a cultural platform for netizens to obtain and exchange information. Since users on the Douban platform are relatively free to discuss different topics, the platform is filled with many unproven rumors; thus, netizens are faced with false information when searching for information. Then, Douban is a suitable research object to explore the phenomena that occur when netizens obtain health-related information on platforms. To explore the truth decay trend when netizens obtain health-related information on domestic social platforms, this study used “COVID-19” as the keyword to conduct a topic search in the Douban group on April 22, 2021. Because vaccine injections were mainly conducted in December 2020, the selected research time span was from December 2020 to April 2021. We selected and discussed posts related to “opinions and thoughts on COVID-19 vaccination” and used the *Octopus* crawler to crawl the main content of the posts and the users' interactive information under the topic. A total of 19 topic contents and 5,665 users' interactions were obtained.

RETRACTED

We stored users' ID, comment time, comment likes, and comment content in a spreadsheet according to different topics. Then, we conducted opinion analysis based on the text's comment content. This part of the work first used regular expressions to clean the symbols (such as @, punctuation, and invalid words), blank information, and emoticons in the comments. Then, based on the opinion mining model established above, the comments were classified according to users' attitudes. We gathered 5,665 attitude distributions for the netizens' comments.

## 4. Research Results

### 4.1. Dynamic Analysis of Netizens' Views and Attitudes

Since the posting time span of the entire topic discussion was from December 2020 to April 2021, for a total of five months, the opinions of netizens were likely to change over time. Thus, we judged the opinions and attitudes of netizens according to the time sequence of posting. The distribution of the netizens' comments of different opinions and positions over time is shown in Figure 2.

Figure 2 shows the evolution of the content of netizens' comments over the changing events. We divided public opinion dissemination periods on the development of topics related to the issue of “COVID-19 vaccination” in accordance with the changes in netizens' different opinions. The first stage was the negative stance period (A: from December 7, 2020, to January 15, 2021), during which netizens held more negative opinions about vaccination, and the number of negative opinions on January 15 peaked (429), accounting for 44% of all comments. The second stage was the period of volatility (B: between January 21 and March 18, 2021), during which the opinions of netizens changed from time to time. On March 3 and 18, netizens' opinions were far more negative than positive, while netizens' positive opinions were dominant on the other five days. The third stage was the positive period (C: from March 24 to April 11). On March 24, 65% of netizens supported the COVID-19 vaccination, and the number of positive opinions reached 405; we found that up to March 31, netizens had held more positive than negative opinions. Although the number of negative opinions on April 11 was 85, the difference in the number of negative and positive opinions was not large (only nine). The figure also shows that when the number of neutral opinions reached the highest number, the number of negative opinions also did (on January 15), and the reverse was true as well. Thus, there is a linear relationship between the neutral and negative opinions of netizens.

RETRACTED

Initially, the netizens' change instance shows that their attitude toward “whether to vaccinate” changed from negative to positive over time and that this change may have been led by the media propaganda and related policies in this period. However, the special case of change in attitude on April 11 and the netizens' reaction during the period of stance fluctuations indicate that other factors affected their attitudes and positions. To explore other factors that affect netizens' stance changes when obtaining health information on social network platforms, we conduct a further analysis by commenting on users' information behavior and on the content of posts.

### 4.2. Stance Analysis Based on User Information Behavior

With the continuous development of social platforms and Internet technology, these platforms have become an important way for netizens to obtain and master the latest information. Netizens can play an important role in sharing information on platforms and expressing it in the form of information behavior (such as information utilization behavior, information interaction behavior, and information reception behavior). These behaviors provide the basis for corresponding research on social platforms. To further explore the factors of change in netizens' positions, the study analyzes the interactive behaviors in user comments on the Douban platform and then analyzes the sum of the number of likes by other users in 19 tweets according to expressing different positions. The distribution is shown in Figure 3.

Figure 3 shows that the interactive behavior of users under different attitudes was also constantly changing. Combined with the changes in the netizens' number of comment positions in Figure 1, it was found that the users' interactive behavior was consistent with this change; that is, when users held mostly negative opinions, they were more inclined to praise the negative comments when browsing a topic. When the users' entire discussion tended to be positive, netizens were more willing to praise the positive position. In addition, there is a certain linear relationship between netizens' neutral views and negative views, and their trends are almost the same. It is worth noting that there were not many neutral views of netizens as a whole, but the number of likes of neutral comments was large. For some posts (e.g., 3 and 10), the number of likes of neutral views exceeded that of positive and negative views. Calculating the interaction index of netizens in the overall event, we found that the cumulative number of neutral views was 27,430, accounting for 35.6% of the total number of likes. Negative views accounted for 34.8%, and the cumulative number of positive views received was 20,573, accounting for only 29.6%. This shows that netizens had more neutral and negative views on the “vaccination dispute”; it was probably because some netizens with neutral and negative attitudes were more willing to reflect their information behavior in the form of likes on social platforms.

RETRACTED

The user's name and type, the number of post interactions, and other information were also counted as part of the user's information behavior. Because the same user nickname was allowed on the Douban platform, we ranked the 19 tweets with a large number of comments (≥8) and the number of likes to explore user interaction regarding the topic of a possible COVID-19 vaccination. The top 15 user IDs were extracted, and the results are shown in Tables 1 and 2.

Tables 1 and 2 describe user information with user information behaviors (likes, comments). The study found that users who posted the most comments (22) received only 16 likes, but those who posted one comment may also get a high number of likes. This phenomenon indicates that the number of comments posted by netizens may not be able to capture the opinions of others. In addition, among the abovementioned multiple user comments, there are many cases where netizens participate in interactions in multiple topic posts (indicated in red, bold numbers). The study found that among the 36 users mentioned above, 10 interacted on multiple topics, five had always held positive views, and three users had always held negative views. Only two users' opinions changed from negative to neutral and from neutral to negative, which shows that in the discussion of the entire topic, about 28% of netizens will continue to participate and express their views. The research found that the opinions of netizens will not change easily, and only a small number of them fluctuate between neutral and negative; this may also be the cause of the linear relationship between netizens' neutral and negative opinions. The research also analyzed different user types, showing that some of the most active users had created posts on this topic. Except for the user whose ID is 186964097, the number of likes received by the rest of the hosts is extremely low (not more than 100). Thus, the host did not play the role of opinion leader in the process of disseminating information about the topic, and users were likely to only post their personal opinions on the issues raised by them.

### 4.3. Position Analysis Based on Topic Content

Judging from the above results, the number of likes received by netizens' comments is not directly related to the number of comments posted by users and whether they are the host or not, and the viewpoints of netizens will not change easily. We selected 14 users with more than 1,000 likes as opinion leaders in this event and extracted their published comments; key topic words in comments with the largest number of likes were extracted according to their different positions. Combining the number of times users mentioned the above keywords under positive, negative, and neutral positions, we further explored the distribution of news that netizens are concerned about from their different positions. The calculation result is shown in Figure 4.

RETRACTED

Figure 4 shows the distribution of topics discussed by 14 opinion leaders from three different positions as well as the main high-frequency words discussed by netizens on different topics. The discussion of topics facing a negative attitude has the highest number of opinions, with a total of six kinds. The main attitudes convey the idea that the vaccine is “not yet mature and will have many side effects,” “the validity period of only six months is too short,” “clinical trials are only going into phase three,” “other vaccines are being used, or I have a fear of any vaccine,” “the current method for controlling the situation in China is safer, so I think it is unnecessary to be vaccinated,” and “I have relevant medical history, and it is not convenient for me to be injected with vaccines.” The high-frequency words of users with negative attitudes are subjective, such as “feeling,” “sensibility,” “unwilling,” and “sense,” showing that most of them are accustomed to making speeches based on their own experience or ideas. Research has found that many netizens with negative attitudes will continue to publish comments such as “the validity period of six months is too short” and “there is no need to vaccinate” for users' opinions that the “validity period is only half a year.” In comments reflecting the positive view, the words “injected,” “already,” and “vaccinated” have high frequency, indicating that netizens who have been vaccinated are more inclined to make corresponding suggestions based on their own experience. The main attitudes of this positive view are “The vaccine has no side effects or the side effects are small,” “the country currently implements free vaccination,” “the sample size of injections is already large,” “the vaccine is an inactivated vaccine and thus very safe,” and “everyone meets the requirements. People with conditions should be vaccinated to achieve herd immunity.” It can be seen that netizens with positive opinions will refute the side effects raised by those with negative opinions, but this kind of refutation has little effect on users holding such negative views. Although the COVID-19 vaccination's supposed validity of six months has already been labeled as fake news, netizens still consume content that they believe in or that is beneficial to their opinions based on their first thoughts.

RETRACTED

In addition, although the opinions of netizens with neutral views are relatively unique (“Vaccination is a personal choice and everyone should take care of their own affairs”), netizens with a neutral attitude are more likely to be recognized by other netizens. This is probably because, in addition to netizens with neutral attitudes who will like their comments, users with negative attitudes will also recognize this type of neutral speech; thus, this may also lead to the number of information behaviors between negative attitudes and neutral attitudes and their linear relationship. Among the 19 posts, one post (March 31) included a poll on whether to get vaccinated or not, and in which 1,769 people participated. The result is shown in Figure 5.

Combining the research results in the previous article, we found that the number of comments from netizens with positive views in the post on March 31 was more than the number of comments with negative views. However, the voting results in Figure 4 showed that 53% of users have not received the COVID-19 vaccine, and 6% chose the option of the onlooker, which shows that in the existing online social platforms, the real-name system required by the network can limit negative speech. It is true that some Internet users do not express their opinions in the form of words, and some have a “seeing the excitement” mentality about related events. At present, the level of information on online platforms is uneven, and the boundaries between opinions and facts have blurred; therefore, many netizens may also be confused about facts and opinions when browsing the news. When a certain point of view contributes to the establishment of their own ideas, netizens will choose to actively agree with it. On the contrary, although the platform will present some facts, when this is contrary to the netizen's thoughts or opinions, the netizen will think that this fact is wrong and ignore it. As a result, some netizens hold an attitude of onlookers in the process of obtaining information and merely look at the posts on the online platform as a pastime.

## 5. Discussion

To explore the related phenomenon of users' access to the health information on social media platforms, our research considers the topic of “whether to get a COVID-19 vaccination” on the Douban platform as an example, exploring the influence of different post topic keywords and user information behavior on the changes of netizens' views and positions. From the above results, we derive the following conclusions.

RETRACTED

### 5.1. Achievements Related to Netizens' Opinion Mining

#### 5.1.1. Benefits of the Analytical Method of Opinion Mining

As suggested by prior research, the analysis of the emotional polarity and different attitudes of netizens on social platforms can be effectively processed through the analysis of netizens' text information [22–24]. This research built a mining dictionary from both positive and negative perspectives based on netizens' views on the COVID-19 vaccine controversy, calculating the opinion and attitude score of netizens based on the formula. According to the scores, the attitudes of netizens were divided into three perspectives: a positive attitude (support vaccination), negative attitude (against vaccination), and neutral attitude (no obvious attitude tendency). The study found that the overall attitude of netizens has changed from a negative stance to a positive stance.

We found that a linear relationship existed between the negative and neutral attitudes of netizens on social network platforms and that their different opinions varied randomly with the passing of time. The number of likes shows that when the position of a topic post tended to be positive, netizens had a tendency to praise the positive comments; conversely, when the position tended to be negative, netizens tended to praise the negative comments. However, in terms of the overall number, the number of Internet users who agree with neutral positions is the highest, and the total number of negative positions is also higher than that of positive positions. It shows that users with negative and neutral positions are more likely to interact with other information behaviors except comments (see Figures 2 and 4). The number of netizens' neutral positions and the change of their likes increase or decrease with the negative positions (see Figures 1 and 2); in addition, the neutral position of netizens was praised more. This result shows that negative attitude netizens may also like the comments of neutral users, and they are more likely to agree with the comments of neutral users (see Figure 3).

#### 5.1.2. Benefits of Social Platforms to Find Changes in Users' Attitudes

The opinions of netizens on social platforms will not change easily. The analysis found that when netizens pay attention to a hot topic, they will not only track and reply to a post but also interact with posts on other related topics. However, during the entire process of posting an article, netizens will not easily change their position, and they may only sway between negative and neutral views (Tables 1 and 2). As there is a certain “fake news” environment on social platforms, netizens may be confused about facts and opinions. Therefore, when a piece of information that contradicts one's opinion is generated on a social platform, netizens will not immediately confirm its authenticity and will often mistake facts for the personal opinions of a certain netizen, thereby ignoring them. This result shows that netizens tend to agree with information similar to their own opinions on social platforms and will not further analyze its authenticity, or a small group of them simply ignores any other news and only believes their own personal opinions. This behavior is also a trend of truth decay on social networking platforms.

RETRACTED

Exploring the different attitudes and stance changes of netizens on social platforms, combining the user's information behavior and the topic content of the posts, allows us to explore phenomena that occur when users obtain health information on social platforms. The relevant conclusions drawn can provide ideas for subsequent research on the acquisition of health information on social platforms. They may help relevant platforms and departments better understand the phenomenon of information decline in social platforms, respond effectively to the questions raised by users on the platform, and publish more authentic and effective tweets for users to relieve pressure from the information on the platform. The information behavior of Internet users should be diverted to control the negative comments of netizens, fundamentally cutting rumors at the source as well as their channels of transmission. It can provide suggestions for the government and related enterprises to deal with the release and dissemination of health information on social platforms and effectively improve the utilization rate of online users to obtain such information.

### 5.2. Users' Information Behavior

Users' information behavior [25, 26] (especially likes, comments, and so on [27, 28]) can convey their effective participation in social platforms. This study first divided the attitudes of netizens according to the time series distribution and found that when netizens' emotions tended to be negative, the number of likes in negative comments also increased at the same time. Netizens with neutral and negative attitudes are more willing to reflect their information behavior in the form of likes on social platforms, and the changes of the two attitudes have a linear relationship. Opinion leaders also play an important role on social platforms [29]. However, the study found that the creator of the post was not an opinion leader, and the number of likes received by netizens' comments has nothing to do with the number of comments posted by users and whether they are the host or not; further, netizens' views and positions will not change easily.

RETRACTED

This study combined analyzing high-frequency topic words in the posts of netizens and exploring the distribution of different topics based on three different attitudes. It was found that the main topics discussed by netizens can be explored by analyzing the content of their comments in previous related studies [30, 31]. The number of topics with negative views was the highest, and the number of topics with neutral views was the lowest. Netizens were more inclined to hold subjective language when expressing their opinions and attitudes, and their opinions on social platforms would not change easily.

### 5.3. Truth Decay on Social Media Platform of China

In previous studies, much had been written about rumors [32–34], misinformation or disinformation [35–37], and analysis between facts and truth [38]. The RAND Corporation of the United States released a research report on truth decay, and dozens of introductions and research articles published subsequently abandoned the post-truth theory, overturning its various assumptions. Truth decay defines and describes the four characteristics of the phenomenon. Under this trend, there is an increasing number of fact-related opinions or opinions in the information space that may overwhelm facts; thus, opinions and facts on social media platforms are completely out of balance.

This research combined the relevant trends and phenomena of truth decay to explore the domestic Douban platform and found that netizens tend to hold subjective language when expressing their opinions and attitudes. When netizens comment on their positions, they post some topical keywords that represent their positions. The distribution of opinion leader topics and high-frequency words of netizens shows that users with negative opinions advance six rebuttal topics when expressing them. Moreover, netizens sometimes use subjective words such as “feeling,” “not wanting,” “unwilling,” and “feeling” (see Figure 3). When expressing opinions, users with positive views will also use subjective vocabulary such as “hit,” “already,” and other words that are rich in their own experience. When users with neutral views express their opinions, words such as “whatever” also indicate that they will not rely on official discourse to force others; thus, neutral views are more likely to be accepted by users with negative views. This result shows that when people express opinions on social platforms, they reject facts and data to a certain extent, and they are more inclined to express their opinions based on their own experiences or anecdotes. Therefore, when there are differences between different opinions, the process of gathering opinions will also present differences, which leads to truth decay.

RETRACTED

## 6. Conclusion

This article used the domestic Douban platform as an example to analyze the health information acquisition data related to the “vaccine dispute.” All popular topic posts during December 2020 and April 2021 were collected for further analysis. As netizens paid more attention to the topic of vaccines, the number of comments on each post was relatively average. Through the above research, it was found that the attitude of netizens changed from more negative attitude to more positive attitude with the development of events, and their attitudes fluctuated until they finally tended to be more positive. However, Internet users would not easily change their original views and ideas. The development of the Internet and social media not only promotes but also facilitates the spread of false information. As far as the vaccination dispute is concerned, netizens advance their own views on a controversial event, and when browsing other people's views, they accept their own according to their own preferences and interests, even if the news is a rumor. As a result, social media platforms gather all kinds of views, and the boundaries between facts and opinions will gradually blur. Netizens will selectively block the truth that they should believe but further spread false information, resulting in truth decay on social media platforms.

This research also presents some limitations. Although the case analysis based on the single platform Douban is representative, it can only be used as an exploration to analyze the phenomenon of health information acquisition based on domestic social platforms. Future studies should examine other platforms, combining more platform data for deeper analysis. Future research work will select more platform data to explore user information behaviors in different types of online social platforms and more comprehensively examine and reveal the performance of the truth decay phenomenon on related platforms, with a view to put forward more reference suggestions to promote the development and construction of the platform.

## Figures and Tables

**Figure 1:** Research framework.

**Figure 2:** Netizens' changes in commentary stance over time.

**Figure 3:** Distribution of Internet users' interactive behavior under different positions.

**Figure 4:** Topics of opinion leaders and distribution of high-frequency words of netizens. (a) Positive attitude, (b) neutral attitude, and (c) negative attitude.

RETRACTED

**Figure 5:** Voting results on the topic of vaccinations.

**Table 1:** Description of user information with many comments.

User's ID	Number	User's type	User's attitude
175613859	22	Original poster	Negative attitude (16)
197373778	20	Original poster	Negative attitude (56)
108840752	17	General user	Negative attitude (2,647)
122904147	13	Original poster	Neutral attitude (17)
134521287	**13**	General user	Positive attitude (557)
54804762	12	General user	Positive attitude (103)
179536118	**11**	General user	Negative attitude (9)
147110811	10	General user	Negative attitude (19)
186964097	10	Original poster	Neutral attitude (3 349)
191986687	10	General user	Positive attitude (1)
28990561	**10**	General user	Positive attitude (38)
VALLA	**10**	General user	Positive attitude (65)
160648681	9	General user	Positive attitude (120)
3044425	**9**	General user	**Neutral turn to negative attitude** (**27**)
107117165	8	General user	Negative attitude (30)
133641969	8	General user	Positive attitude (26)
173384722	**8**	General user	Negative attitude (0)
213154669	8	General user	Negative attitude (16)
3324220	**8**	General user	Positive attitude (49)
69911308	**8**	General user	Positive attitude (41)
whitedwarf000	8	Original poster	Neutral attitude (31)

**Table 2:** Description of user information with many likes.

User's ID	Number	User's type	User's attitude
iMa7ch	2	General user	Neutral attitude (4,456)
182565704	2	General user	Neutral attitude (2,687)
174862143	1	General user	Negative attitude (2,649)
167296657	**3**	General user	**Negative attitude turn to neutral attitude** (**2,205**)
80573402	1	General user	Negative attitude (1,884)
gardenia_v	1	General user	Negative attitude (1,815)
55283261	1	General user	Positive attitude (1,651)
Woailongkuan	1	General user	Positive attitude (1,566)
74633635	1	General user	Positive attitude (1,414)
64195031	2	General user	Neutral attitude (1,238)
Trista55	**2**	General user	Negative attitude (1,156)
134521287	3	General user	Positive attitude (1,024)
Freut-mich	2	General user	Positive attitude (846)
214305228	1	General user	Neutral attitude (815)
144794436	2	General user	Neutral attitude (779)

^∗^Note that the number in brackets indicates the number of likes.

## Data Availability

The data of users' behavior of health-related information about “vaccine injection” in Douban are available at https://www.douban.com/group/topic/.
